# A De Novo Transcriptome Analysis Identifies Cold-Responsive Genes in the Seeds of *Taxillus chinensis* (DC.) Danser

**DOI:** 10.1155/2022/9247169

**Published:** 2022-07-06

**Authors:** Jine Fu, Lingyun Wan, Lisha Song, Lili He, Ni Jiang, Hairong Long, Juan Huo, Xiaowen Ji, Fengyun Hu, Shugen Wei, Limei Pan

**Affiliations:** ^1^Guangxi Botanical Garden of Medicinal Plants, Nanning 530023, China; ^2^Guangxi Key Laboratory for High-Quality Formation and Utilization of Dao-di Herbs, China

## Abstract

*Taxillus chinensis* (DC.) Danser, a parasitic plant of the *Loranthaceae* family, grows by attacking other plants. It has a long history of being used in Chinese medicine to treat multiple chronic diseases. We previously observed that *T. chinensis* seeds are sensitive to cold. In this study, we performed transcriptome sequencing for *T. chinensis* seeds treated by cold (0°C) for 0 h, 12 h, 24 h, and 36 h. TRINITY assembled 257,870 transcripts from 223,512 genes. The GC content and N50 were calculated as 42.29% and 1,368, respectively. Then, we identified 42,183 CDSs and 35,268 likely proteins in the assembled transcriptome, which contained 1,622 signal peptides and 6,795 transmembrane domains. Next, we identified 17,217 genes (FPKM > 5) and 2,333 differentially expressed genes (DEGs) in *T. chinensis* seeds under cold stress. The MAPK pathway, as an early cold response, was significantly enriched by the DEGs in the *T. chinensis* seeds after 24 h of cold treatment. Known cold-responsive genes encoding abscisic acid-associated, aquaporin, C-repeat binding factor (CBF), cold-regulated protein, heat shock protein, protein kinase, ribosomal protein, transcription factor (TF), zinc finger protein, and ubiquitin were deregulated in the *T. chinensis* seeds under cold stress. Notably, the upregulation of CBF gene might be the consequences of the downregulation of MYB and GATA TFs. Additionally, we identified that genes encoding CDC20, YLS9, EXORDIUM, and AUX1 and wound-responsive family protein might be related to novel mechanisms of *T. chinensis* seeds exposed to cold. This study is first to report the differential transcriptional induction in *T. chinensis* seeds under cold stress. It will improve our understanding of parasitic plants in response to cold and provide a valuable resource for future studies.

## 1. Introduction

*Taxillus chinensis* (DC.) Danser, also named “Sang Ji Sheng,” is a parasitic plant from the *Loranthaceae* family and grows by attacking other plants, such as *Aceraceae*, *Anacardiaceae*, *Euphorbiaceae*, *Fabaceae*, *Fagaceae*, *Juglandaceae*, *Moraceae*, *Rosaceae*, and *Rutaceae* [1]. Because the leaves and stems of *T. chinensis* have been used to treat angina pectoris, arrhythmia, hypertension, rheumatism, stroke, and threatened abortion [1], it has a long history of being used in the Chinese medicine. It is mainly distributed in the southern and southwestern areas of China, probably due to the warm and humid climate. Our knowledge of *T. chinensis* is very limited, especially its responses to abiotic stresses.

Among the abiotic stresses, temperature is an important factor that affects the plant physiological processes [2]. Cold stress, including chilling (<20°C) and freezing (<0°C), exerts a substantial effect on the plant health and potentially limits the plant growth, development, yield, and geographical distribution [3]. As a mechanism to combat low environmental temperature, plants have developed a series of response mechanisms to adjust gene expression and further to enhance their cold tolerance [4]. In recent decades, many studies have been elucidated the molecular mechanisms involved in the plant cold acclimation. CBF/DREB- (C-repeat binding factors/dehydration factor/dehydration responsive element binding factor-) dependent signalling was characterized as a key and conserved regulatory mechanism of many plants in response to cold, together with the CBF activators (e.g., ICE1, CAMTA3, and BZR1/BES1) and repressors (e.g., MYB15, PIFs, and EIN3) [5, 6]. By binding to the cis-acting elements, CBFs induce the expression of numerous downstream cold-responsive (COR) genes [3]. Upon the exposure to cold, some protective genes are transcribed to enhance the cold tolerance of plants, such as heat shock proteins (HSPs) [7], protein kinases (PKs; e.g., SNF1-related protein kinases 2.6/open stomata 1) [8], cryoprotective proteins [4], zinc finger proteins [6], and various metabolites [9]. Additionally, many transcription factors (TFs) have been reported to regulating gene expression in plants under cold stress, such as ethylene response factors [10], NACs [11], MYBs [12], bHLHs [13], and WRKYs [14]. In addition, CBF-independent regulatory pathways have also been characterized in plants to enhance their cold tolerance, including the plant hormones auxin, abscisic acid, ethylene, gibberellins, and jasmonic acid [15]. However, little is known about the molecular mechanisms activated in *T. chinensis* seeds in response to cold.

Transcriptome sequencing, a next-generation sequencing technology, is an efficient method to detect gene expression profiles and elucidate the breadth of molecular mechanisms involved in many physiological processes [16]. It has been widely used to identify key genes and factors involved in the responses to abiotic/biotic stresses in plants due to its advantages in the large-scale functional assignment of genes, thorough qualitative and quantitative analyses of gene expression, improved sensitivity, and accurate profiling of eukaryotic transcriptomes for both model and nonmodel organisms [17, 18]. Importantly, it facilitates analyses of gene expression in organisms whose genomes are not accessible. For example, using transcriptome sequencing and de novo assembly analysis, Liu et al. investigated the transcriptome of *Rumex patientia* during cold stress and identified 66 genes that are putatively involved in the response to cold stress, including members of the MYB, AP2/ERF, CBF, Znf, bZIP, NAC, and COR families [19]. Mohamed Sathik et al. employed transcriptome sequencing to study abiotic stress responsive genes in *Hevea brasiliensis* [20]. Fu et al. analyzed the transcriptome of Elymus nutans under cold stress and identified 26 hub genes playing a central role in the response to cold [21]. Similar to these studies, transcriptome sequencing technology will enable us to study changes in gene expression changes in *T. chinensis* seeds under cold stress.

Previously, our lab identified genes that are expressed in response to water loss in *T. chinensis* seeds [22], such as RD22, HSP, and various TFs (MYB, WRKY, and ethylene-responsive transcription factors), and reported the regulatory miRNAs in *T. chinensis* seeds in response to cold [23], such as miR408, miR393b, miR946, ath-miR779.2, miR398, and miR9662. Interestingly, ICE3, IAA13, and multiple TFs (e.g., WRKY and CRF4 and TCP4) were shown to be targets of the dysregulated miRNAs identified in the *T. chinensis* seeds under cold stress [23]. In the present study, we used the same material as the miRNA study and investigated changes in gene expression changes in *T. chinensis* seeds in response to cold using transcriptome sequencing technology. This study is the first to analyze the changes in gene expression in *T. chinensis* seeds under cold stress, and our results will improve our understanding of molecular mechanisms of cold stress in *T. chinensis* seeds.

## 2. Materials and Methods

### 2.1. Sample Collection and Cold Treatment

The original seeds of *T. chinensis* were obtained from three mulberry trees in the wild, and no permissions were required to collect these samples. The seeds were then confirmed by a senior botanist and deposited in the herbarium of Guangxi Botanical Garden of Medicinal Plants (acc. S0001794). For the cold treatment experiment, we selected 300 *T. chinensis* seeds with similar appearances, including sizes, weights, and health conditions. We observed that the *T. chinensis* seeds were sensitive to temperature and that 0°C was a suitable temperature to study the cold-responsive genes [23]. The seeds were divided into three groups—no treatment (A0) and cold treatment for 12 h (A1), 24 h (A2), and 36 h (A3). Then, we examined the viability of A0, A1, A2, and A3 by immersing the seeds in a solution of 1% (*w*/*v*) 2,3,5-triphenyl tetrazolium chloride (TTC, Sigma), as previously described [22].

### 2.2. Total RNA Isolation, cDNA Library Construction, and Deep Sequencing

Total RNA was extracted from the *T. chinensis* seeds (100 mg) exposed to cold for 0 h (A0), 12 h (A1), 24 h (A2), and 36 h (A3) using TRIzol reagent, as previously described [22]. Next, an Agilent 2100 Bioanalyzer (Agilent Technologies) was used to determine the quantity and quality of the total RNA. Equal amounts of total RNA (1 *μ*g) were used to construct the cDNA libraries for transcriptome sequencing. Briefly, mRNAs were enriched with magnetic oligo (dT) beads and fragmented into ~200 bp fragments, followed by the double strand cDNA library construction using random hexamer N6 primers. Next, the double strand cDNA libraries were end repaired by adding a phosphate at the 5′-end and sticky “A” to the 3′-end. After the sequencing primers were ligated to each library and multiple libraries were pooled using the index technology, the pooled library was sequenced on the BGISEQ-500 RS platform with a paired-end 150 (PE150) strategy at BGI-Shenzhen.

### 2.3. Read Cleaning and De Novo Assembly of the Transcriptome

Raw reads were processed using SOAPnuke to remove the low-quality reads, reads with adaptors, and contaminating reads [24]. The obtained clean reads were quality controlled using FASTQC, as previously described [25]. Then, the clean reads of all samples assembled into the transcriptome using the TRINITY software with default parameters, according to a published protocol [26]. We next aligned all the clean reads to the assembled transcriptome using Bowtie2 and determined the global gene expression profile using the RSEM (RNA-Seq by Expectation-Maximization) method [27, 28]. The fragments per million reads per kilo base mapped (FPKM) method was used to normalize gene expression. We filtered genes expressed at low levels (FPKM < 1) from the assembled transcriptome for quality control of the assembled transcriptome. CD-HIT was used to cluster the assembled *T. chinensis* genes [29]. BUSCO was used to evaluate the completeness of the assembled transcriptome [30].

### 2.4. Transcriptome Annotation

We annotated the assembled *T. chinensis* transcriptome by mapping it to public databases. In detail, the transcriptome was aligned to the NT database using BLASTn and aligned to the COG, KEGG, NR, and SwissProt databases using BLASTx. Then, open reading frames (ORFs) were predicted in the assembled transcriptome and aligned to the InterPro database using InterProScan. Gene Ontology annotations were retrieved from the mapping results of InterPro and NR. KEGG pathway annotation results were retrieved from the KEGG pathway mapping results. In combination with the BLAST results, we fetched the possible coding sequence (CDS) regions in the assembled transcriptome. Likely proteins encoded by the assembled transcriptome were predicted by TransDecoder and were used to identify signal peptides and transmembrane helices with SignalP (v5.0b) and TMHMM (v2.0c), respectively, according to the manufacturers' protocols.

### 2.5. Gene Expression Profile and Differential Expression Analysis

We aligned the clean reads of each sample to the assembled transcriptome using Bowtie2 to profile gene expression in the *T. chinensis* seeds under cold stress [27]. Then, the RSEM method was used to count the reads aligned to each gene and normalize the gene expression using the FPKM method [28]. We used edgeR to calculate the *p* values and false discovery rate (FDR) to identify differentially expressed genes in the *T. chinensis* seeds under cold stress. Some cut-offs were used to identify the DEGs, including log2 fold change (log2FC) > 1 or < -1, *p* value < 0.05, coefficient of variation (CV) < 0.7, and false discovery rate (FDR) < 0.1.

### 2.6. Functional Analysis

Using the GO and KEGG pathway annotations for the assembled *T. chinensis* seed transcriptome, we analyzed the enriched GO terms (biological processes, molecular functions, and cellular components) and KEGG pathways of the DEGs. Initially, *p* values were calculated using the Fisher's exact test to show the significance, and *q* values were calculated using the R package “qvalue” for quality control of the *p* values.

### 2.7. qRT-PCR

We selected 11 genes for qRT-PCR validation, and 18S rRNA was used as an internal control. Forward and reverse primers were predicted using Primer3 and synthesized at BGI (Shenzhen) (Table S1). The procedure for the qRT-PCR experiment was the same as that in our previous study [22]. Then, we calculated the ΔCt value to determine the expression levels of target genes in a sample and ΔΔCt value to assess the difference in gene expression between two samples. We used relative normalized expression (RNE) to show the gene expression changes: RNE = 2^−∆∆Ct^ and calculated its log2 value (log2RNE) to compare the changes in gene expression identified using RNA-Seq and qRT-PCR.

## 3. Results

### 3.1. Overview of Deep Sequencing Results and De Novo Assembly

We previously observed that *T. chinensis* seeds were sensitive to temperature and that 0°C was a suitable temperature to study the cold responsive genes in *T. chinensis* seeds [23]. Thus, we performed paired-end transcriptome sequencing in triplicate for *T. chinensis* seeds exposed to 0°C for 0 h (A0), 12 h (A1), 24 h (A2), and 36 h (A3). Initially, we obtained 728.82 million raw reads and 725.59 million clean reads after data cleaning. Then, the clean reads of all samples were merged and used for the de novo assembly and analysis. TRINITY assembled 257,870 transcripts derived from 223,512 genes. After the expression levels of the assembled genes were estimated, we filtered genes at low levels (FPKM < 1) from the assembled transcriptome and clustered the genes. Finally, we obtained 111,390 transcripts corresponding to 98,514 *T. chinensis* genes. The statistical values of the assembled transcriptome are shown in Table 1. The GC content and N50, a statistical measure of the average length of a sequence set, were calculated as 42.29% and 1,368, respectively, for the assembled *T. chinensis* transcriptome. Next, we evaluated the length distribution of the assembled *T. chinensis* transcriptome. As shown in Figure 1(a), 39,302 transcripts (39.89%) with lengths between 200 and 300 nt and 3,341 transcripts (1.25%) longer than 4,000 nt were obtained. The completeness of the assembled *T. chinensis* transcriptome was evaluated using BUSCO, which identified 249 (97.7%) complete (197 complete and single-copy and 52 complete and duplicated), 4 fragmented, and 2 missing BUSCOs.

### 3.2. Annotation of the Assembled *T. chinensis* Transcriptome

We next annotated the assembled *T. chinensis* transcriptome by mapping it to multiple databases. A total of 59,830 transcripts were annotated, of which 37,643, 52,000, 25,421, 26,725, 16,092, 21,442, and 26,866 were aligned to the NR, NT, SwissProt, KEGG (Kyoto Encyclopedia of Genes and Genomes) pathway, COG (Clusters of Orthologous Groups), GO (Gene Ontology), and InterPro databases, respectively (Figure 1(b)). Notably, 10,509 transcripts were annotated by all these databases (Figure 1(b)). Among the NR mapping results, we found that the top four species hits to the assembled *T. chinensis* transcriptome were *Vitis vinifera* (10,313 transcripts), *Theobroma cacao* (1,980 transcripts), *Nelumbo nucifera* (1,828 transcripts), and *Ziziphus jujuba* (1,481 transcripts) (Figure 1(c)). COG annotation (Figure 1(d)) revealed 1,126, 730, 198, and 31 transcripts from “signal transduction mechanism,” “energy production and conversion,” “defense mechanism,” and “cell motility,” respectively. Among the 26,276 transcripts with GO annotations (Figure 1(e)), we found that the top four GO terms were “metabolic process” (13,530 transcripts), “cellular process” (12,603 transcripts), “catalytic activity” (10,471 transcripts), and “binding” (9,847 transcripts). Additionally, we identified 1,061 and 192 transcripts related to “signaling” and “signal transducer activity,” respectively (Figure 1(e)). By mapping the *T. chinensis* transcriptome to the KEGG pathway database, we identified transcripts from five categories (Figure 1(f)), including cellular processes, environmental information processing, genetic information processing, human diseases, metabolism, and organismal systems. Interestingly, metabolism was enriched in most of the transcripts, and 4,896 transcripts were annotated from the “global and overview maps” of metabolisms. We detected 833 and 855 transcripts involved in the pathways of “signal transduction” and “environmental adaption,” respectively (Figure 1(f)).

Using the BLAST results, we identified 38,479 coding sequences (CDSs) from the assembled *T. chinensis* transcriptome, which consisted of 24.21 million bases (mean length: 629, N50: 927, and GC content: 46.95%). Next, ESTScan identified 3,704 CDSs from the *T. chinensis* transcriptome, whose size was 1.26 million bases (mean length: 339, N50: 330, and GC content: 50.74%) [31]. Thus, in total, we obtained 42,183 CDSs for the *T. chinensis* seeds under cold stress (25.46 million bases, mean length: 603, N50: 891, and GC content: 47.14). Furthermore, we predicted 35,268 likely proteins derived from 30,728 of the *T. chinensis* transcripts using TransDecoder (https://github.com/TransDecoder/TransDecoder). SignalP and TMHMM identified 1,622 signal peptides and 6,795 transmembrane domains among the likely proteins of *T. chinensis* seeds. Annotations obtained from different perspectives improved our understanding of the assembled transcriptome and were useful for the identification of cold-responsive genes in the *T. chinensis* seeds. However, further experiments are required to explore some transcripts that were annotated without encoding capacity.

### 3.3. Gene Expression Profiles of the *T. chinensis* Seeds under Cold Stress

The viability of *T. chinensis* seeds decreased quickly under cold stress, and we investigated the cold-responsive genes of *T. chinensis* seeds. Read mapping showed that 81.52%-84.95% of the clean reads were aligned to the assembled transcriptome. Then, we obtained 17,236 genes with FPKM > 5 in the *T. chinensis* seeds under cold stress, of which 15,414, 14,658, 14,963, and 14,849 were distributed in A0, A1, A2, and A3, respectively (Figure 2(a), Table 1, and Table S2). Pearson's correlation analysis revealed that the linear correlation between these samples was greater than 0.97, indicating a limited difference between them. The distribution of gene expression revealed that 58.30%-58.68% of detected genes in the *T. chinensis* seeds were expressed with FPKM values ranging from 10 to 99 (Figure 2(b)). Notably, 64, 69, 74, and 83 *T. chinensis* genes were expressed at more than 1000 FPKM in A0, A1, A2, and A3, respectively.

We next compared the highly expressed genes in all four samples (Table S2), and 9 of the top 10 highly expressed genes were shared by all four samples. Among them, TR50621|c2_g12 was specific to A0, and TR36565|c1_g1 (lipid transfer protein) was specific to A1, A2, and A3. Then, we counted the numbers of some known cold responsive genes. As shown in Table 2, in the *T. chinensis* seed transcriptome, we identified 18, 22, 3, 9, 36, 529, 327, 402, 82, and 297 genes related to abscisic acid, aquaporin, C-repeat binding factor (CBF), cold stress (e.g., cold-regulated (COR) protein), heat shock protein (HSP), protein kinase (PK), ribosomal protein (RP), transcription factor (TF), zinc finger protein (ZFP), and ubiquitin, respectively.

### 3.4. Differentially Expressed Genes in the *T. chinensis* Seeds under Cold Stress

We next identified differentially expressed genes (DEGs) in the *T. chinensis* seeds under cold stress. Compared to A0, we detected 983 (538 upregulated and 445 downregulated), 451 (315 upregulated and 136 downregulated), and 1,857 (1,101 upregulated and 756 downregulated) DEGs in A1, A2, and A3, respectively (Figure 2(c) and Table S3). As shown in Figure 2(d), DEGs in A1 and A0 were involved in biological processes, including “GO:0009909~regulation of flower development,” “GO:0071840~cellular component organization or biogenesis,” “GO:0006807~nitrogen compound metabolic process,” “GO:0006096 ~ glycolytic process,” “GO:0046037~GMP metabolic process,” and “GO:0009697~salicylic acid biosynthetic process.” However, after 24 h of cold treatment, the DEGs between A2 and A0 were enriched in the biological processes “GO:0006810 ~ transport,” “GO:0008643 ~ carbohydrate transport,” “GO:0071555~cell wall organization,” “GO:0034757~negative regulation of iron ion transport,” and “GO:0034220~ion transmembrane transport” (Figure 2(e)). After 36 h of cold treatment, the DEGs were found to participate in the biological processes such as “GO:0006970~response to osmotic stress,” “GO:0009733~response to auxin,” and “GO:0006281 ~ DNA repair” (Figure 2(f)). Interestingly, cold-responsive genes of *T. chinensis* seeds were found to be enriched in different pathways during the cold treatment. For example, DEGs in A1 and A0 were enriched in 5 KEGG pathways (e.g., “ubiquitin mediated proteolysis,” “plant-pathogen interaction,” “oocyte meiosis,” “glutathione metabolism,” and “cell cycle”) (Figure 2(g)); “MAPK signaling pathway-plant” was triggered by the DEGs in *T. chinensis* seeds after 12 h of cold treatment (Figure 2(h)), and pathways such as “plant-hormone signal transduction,” “oxidative phosphorylation,” and “flavone and flavonol biosynthesis” were initiated in the *T. chinensis* seeds after 36 h of cold treatment (Figure 2(i)). The number of DEGs from different gene families, such as aquaporin, CBF, COR, PK, RP, TF, ZFP, and ubiquitin proteins, is shown in Table 2.

### 3.5. Cold-Responsive Genes in *T. chinensis* Seeds

Prior to identifying early and late cold-responsive genes in *T. chinensis* seeds, we showed the expression levels of all DEGs in these samples (A0, A1, A2, and A3) by constructing a heat map (Figure 3(a)). Venn diagrams (Figure 3(b)) revealed that 231 upregulated and 77 downregulated genes were shared in seeds during the cold treatment for 12 h, 24 h, and 36 h. Among them, 1 aquaporin, 1 ABA-associated gene, 13 HSPs, 12 TFs, 5 ZFPs, and 1 ubiquitin gene were commonly deregulated (Table 2). Notably, among the commonly upregulated genes detected in *T. chinensis* seeds under cold stress, we identified 5, 2, 3, and 3 shared upregulated genes encoding CDC20-1, CDC20-2, YLS9, and EXORDIUM, respectively (Table S3). In addition, 332 (151 upregulated and 181 downregulated) and 1,225 (707 upregulated and 518 downregulated) DEGs were specifically deregulated in *T. chinensis* seeds at the early (A1) and late (A3) stages of cold treatment, respectively (Figure 3(b)). Among the genes that were specifically deregulated in A1, we identified TR43917|c0_g1 encoding a wound-responsive family protein, TR37450|c1_g1 encoding auxin transporter protein 1 (AUX1), and three genes encoding aquaporins (Figure 3(c) and Table S3). These genes might be related to the early response to cold in *T. chinensis* seeds. Among the genes specifically deregulated in A3, we found 11 genes encoding disease resistance proteins, 4 genes encoding ER TFs, TR15040|c0_g1 encoding auxin-responsive protein IAA1-like, TR37606|c0_g4 encoding ethylene receptor, and TR39623|c0_g1 encoding ethylene response factor 10 (ERF10) (Figure 3(c) and Table S3), which might function in the late cold responsive stage in *T. chinensis* seeds.

### 3.6. Transcription Factors

We next further analyzed the TF expression patterns in the *T. chinensis* seeds under cold stress. Four hundred two TF genes were annotated in the *T. chinensis* seed transcriptome (Table 2), and 76 were differentially expressed in response to cold (Table 3). ER TF was the largest (27 genes) class that was differentially expressed in *T. chinensis* seeds under cold stress (Table 3 and Figure 4(a)). Notably, the expression levels of some ER TF genes were increased in the *T. chinensis* seeds at the late stage of cold treatment but not in A1 or A2. The downregulation of ER TF genes might be related to the seed development and other seed activities at normal temperature. Similar to ER TF genes, the functions of some other TF classes, such as WRKY and bHLH, are difficult to determine, as we observed both up- and downregulation of these genes in the *T. chinensis* seeds under cold stress (Figure 4(b)). However, the upregulation of AP2 domain class TF genes and the downregulation of GATA and MYB TF genes might participate in the cold response of the *T. chinensis* seeds, as they showed consistent regulation at all three time points of the *T. chinensis* seeds under cold stress (Table 3 and Figure 4(b)).

### 3.7. Protein Kinases, Ribosomal Proteins, and Zinc Finger Proteins

As shown in Table 2, 60, 11, and 20 genes encoding PK, RP, and ZFP were differentially expressed in the *T. chinensis* seeds under cold stress, and their expression patterns are presented in Figure 4(c). Although some genes encoding calcium dependent, serine-threonine (e.g., LRR receptor-like and PTI1-like tyrosine) PKs were upregulated in A1 compared to A0; more PK genes from these subtypes were upregulated in A3 (Figure 4(c), left). Interestingly, we identified 402 RP genes in the *T. chinensis* seed transcriptome, but only 11 of them were deregulated in response to cold stress, including four 40S (e.g., RPS3 and RPS4) and seven 60S (e.g., RPL6, RPL7, and RPL10) RP genes. The overall expression of RP genes was upregulated in *T. chinensis* seeds to defend against cold stress (Figure 4(c), middle). We also detected both upregulated and downregulated ZFP genes in *T. chinensis* seeds after cold treatment (Figure 4(c), right). Two major classes of ZFP genes were identified and presented divergent expression patterns: dof ZFP and ZAT. The dof ZFP genes were downregulated, while the ZAT genes were upregulated in *T. chinensis* seeds under cold stress.

### 3.8. qRT-PCR

We used qRT-PCR to validate the expression patterns of genes in the *T. chinensis* seeds under cold stress. Eleven genes (e.g., CBF1, GATA4, MYB44, ERF4, ERF010, and ZAT10) and an internal control (18S rRNA) were selected to perform the qRT-PCR validation experiment. The primers for these candidate genes used in qRT-PCR are listed in Table S1. After ∆∆Ct values were calculated, we used log2 relative normalized expression (log2RNE) to show the changes in the expression of target genes between two samples, similar to the transcriptome sequencing. Among the 33 events showing the expression patterns of the target genes in *T. chinensis* seeds under cold stress, we found that 31 (93.9%) exhibited consistent changes in both RNA-Seq and qRT-PCR experiments (Figure 5). Notably, the expression patterns of CBF1, SOBIR1, and ERF10 were confirmed by qRT-PCR. The high agreement of gene expression patterns obtained using RNA-Seq and qRT-PCR indicates that the genes identified in this study might function in the cold response of *T. chinensis* seeds.

## 4. Discussion

*T. chinensis* is a plant that is sensitive to cold, and this study was designed to investigate the changes in gene expression in *T. chinensis* seeds under cold stress. Due to the lack of genome sequences, we assembled the transcriptome for *T. chinensis* seeds using RNA-Seq, similar to the studies of other plants, such as *Magnolia wufengensis* [32], *Passiflora edulis* Sims [33], *Hevea brasiliensis* [20], and *Rumex patientia* [19]. We assembled 98,514 *T. chinensis* genes and 35,268 likely proteins expressed in the *T. chinensis* seeds in response to cold. Interestingly, many of the *T. chinensis* genes were predicted to have similarities with grape genes (Figure 1(c)). A number of cold-responsive genes are involved in multiple biological processes and pathways, such as plant hormone signal transduction [32, 33] and metabolic processes [19, 20, 32, 33]. The DEGs identified in the *T. chinensis* seeds under cold stress were determined to be enriched in these pathways (Figures 2(d)–2(i)). Some known cold-responsive genes, including ABA, aquaporin, CBF, COR, HSP, PK, RP, ZFP ubiquitin, and TFs, were identified (Table 2). In addition, we found that genes encoding CDC20-1, CDC20-2, YLS9, and EXORDIUM were upregulated in the *T. chinensis* seeds in response to cold (Table S3).

Cold acclimation temperatures have the potential to induce profound changes in the plant transcriptome. Approximately 4% to 20% of the genes in the *Arabidopsis* genome are affected by cold [34, 35]. Interestingly, different pathways were activated in the *T. chinensis* seeds during cold treatment (Figures 2(g)–2(i)). The “MAPK signalling pathway–plant” was significantly enriched in the DEGs in A2, but not A1, compared to A0 (Figure 2(h)). This pathway has been reported to modulate plant tolerance to multiple abiotic stresses, such as drought, salt, cold, and heat [36]. The MAPK cascades have been reported to convert the environmental stimuli into cellular responses and to negatively regulate freezing tolerance via the phosphorylation of ICE1, a basic-helix-loop-helix transcription factor that regulates the expression of CBF genes [37], which mediate cold-inducible transcription and play a key role in freezing tolerance and cold acclimation by binding to the C-repeat/DRE element [38]. MAPK pathway activation is a rapid response to cold, as MPK3, MPK4, and MPK6 are rapidly activated after cold treatment [37]. Compared to A0, we identified 10, 14, and 21 genes from the MAPK pathway that were differentially expressed in the *T. chinensis* seeds after exposure to cold for 12 h, 24 h, and 36 h, respectively (Figures 2(h) and 2(i)). Among them, MPK9 was commonly upregulated at all three time points while two MAPKK kinases (NPK1-like and YODA) were specifically upregulated in A3 (Table S3). NPK1-like and its clustered genes, namely, other NPK-like genes (e.g., OsNPKL2, 3, and 4), are induced by cold in rice [39]. YODA was shown to be upstream of MKK4/MKK5, a negative regulator of freezing tolerance [37], and downstream of the ER receptor in regulating coordinated local cell proliferation, which shapes the morphology of plant organs [40].

Interestingly, the ICE1 TF gene (TR144797|c0_g1) was not dysregulated in *T. chinensis* seeds under cold stress; however, the CBF1 gene (TR16191|c0_g1) was upregulated during this process (Table S2). The *Arabidopsis* CBF genes are transcribed within a short period of exposure to cold stress and subsequently induce the COR gene expression [41, 42]. We detected two COR genes that were deregulated in the *T. chinensis* seeds under cold stress: TR39356|c0_g1 (cold-regulated 413 plasma membrane protein 2-like) and TR38199|c0_g1 (cold-regulated gibberellin-regulated protein 1 LTCOR12) (Table S3). In *Arabidopsis*, CBFs were shown to be negatively regulated by a cold-induced C2H2 zinc finger transcription factor gene, ZAT12 [43], which is also regulated by ICE1 [44], and to be inducers of the C2H2 transcription factor gene ZAT10 [45]. In the present study, we observed the upregulation of ZAT10 and the downregulation of ZAT12 (Table S3) in *T. chinensis* seeds under cold stress. CBF2, ZAT12, and ZAT10 were shown to regulate 172, 67, and 54 COR genes in *Arabidopsis* [46]. Thus, the upregulation of CFB and COR genes might be regulated by other modulators, such as MYB15, a negative regulator of CBFs in *Arabidopsis* [47], and GATA TFs, which were observed to be downregulated in *T. chinensis* seeds under cold stress (Figure 4(b)).

LRR-RLK (LRR receptor-like serine/threonine-protein kinase) might be another group of PKs participating in the early response to cold stimuli in *T. chinensis* seeds, as we identified 8 LRR-RLK genes (5, 1, and 5 in A1, A2, and A3, respectively) that were differentially expressed in the *T. chinensis* seeds under cold stress (Figure 4(c) and Table S3). LRR-RLKs are a well-known class of RLKs that play important roles in plant growth, development, hormone perception, and responses to biotic/abiotic stresses [48]. They have been reported to be positive regulators of cold tolerance in *Glycine soja* [48], *Glycine max* [48], and *Oryza sativa* [49]. We also observed 10 aquaporin genes that were upregulated in the *T. chinensis* seeds under cold stress (Table 2 and Table S3). Low environmental temperature has been proven to inhibit water uptake by roots [50]. In chilling-sensitive rice, low temperature treatment resulted in a gradual increase in the expression of aquaporin genes [51]. Li et al. found that the aquaporin gene GhTIP1 was substantially upregulated in cotyledons but downregulated in roots within a few hours after cotton seedlings were exposed to cold [52]. These studies, including the present study, support the hypothesis that aquaporin genes might be involved in the response to cold stress in plants. RP genes might be another class of cold-induced genes in plants that potentially enhances the cold tolerance, as both large and small RP subunits have been shown to be induced in soybean in response to cold [53]. In tobacco, ribosomal proteins Rps2, Rps4, and Rpl20 are essential for cell survival, and Rpl33 is required for sustaining a sufficient plastid translation capacity in cold temperatures [54]. The upregulation of RP genes was also observed in *Hippophae rhamnoides* under cold and freeze stress [55]. In *T. chinensis* seeds, we observed the upregulation of RP genes (Table 2 and Table S3), including RPL36, RPS3, RPS4, and RPS8. However, additional experiments are needed to elucidate the regulatory network of RP genes and their functions in *T. chinensis* seeds under cold stress, along with some other genes, such as CDC20, YLS9, EXORDIUM, AUX1, and TR43917|c0_g1 (wound-responsive family protein).

## 5. Conclusions

In conclusion, we investigated the transcriptome of *T. chinensis* seeds in response to cold stress. The MAPK pathway might participate in the early response to cold, and the upregulation of CBF genes might be mediated by other regulators, such as MYB and GATA TFs, rather than ICE1. The deregulation of the RP genes, CDC20, YLS9, EXORDIUM, and AUX1, might be a novel mechanisms activated in *T. chinensis* seeds in response to cold. This transcriptome study is the first to analyze *T. chinensis* seeds under cold stress. The results will improve our understanding of mechanisms regulating gene expression in plants under cold stress. More importantly, the results from this study will provide a valuable resource for future studies of *T. chinensis* and benefit the breeding program of *T. chinensis*.

## Figures and Tables

**Figure 1:** *De novo* assembly transcriptome of *T. chinensis* seeds under cold stress and its annotation. (a) Length distribution of transcripts assembled for the *T. chinensis* seeds under cold stress. (b) Numbers of transcripts aligned to different known databases. (c) Number of transcripts aligned to genes from different species in NR. (d) COG function classification of the assembled transcriptome. (e) Gene Ontology annotation for the assembled transcriptome. (f) KEGG pathway annotation for the assembled transcriptome.

**Figure 2:** Gene expression profiles and differential expression analysis for the *T. chinensis* seeds under cold stress. (a) Venn diagram of genes identified in *T. chinensis* seeds in responsive to cold. (b) Distribution of *T. chinensis* genes from different expression levels. (c) Numbers of differentially expressed genes identified in *T. chinensis* seeds under cold stress. Biological processes involved by the DEGs identified in A1 (d), A2 (e), and A3 (f) compared to A0. KEGG pathway enrichment analysis of DEGs identified in A1 (g), A2 (h), and A3 (i) compared to A0.

**Figure 3:** Differentially expressed genes in *T. chinensis* seeds exposed to cold. (a) Heat map of all DEGs identified in this study. (b) Venn diagram of DEGs identified in A1, A2, and A3 compared to A0. (c) Specifically upregulated genes *T. chinensis* seeds in response to cold at early and late stages.

**Figure 4:** Expression patterns of some important gene families in *T. chinensis* seeds under cold stress. (a) Heat map of ER TF genes in *T. chinensis* seeds under cold stress. (b) Heat map of AP2, bHLH, GATA, MYB, and WRKY TF genes in *T. chinensis* seeds under cold stress. (c) Heat maps of protein kinase (left), ribosomal protein (middle), and zinc finger protein (right) genes in *T. chinensis* seeds under cold stress.

**Figure 5:** qRT-PCR validation.

**Table 1:** Overview of transcriptome sequencing and de novo assembly of the T. chinensis seeds under cold stress.

	A0			A1			A2			A3		
	A0_R1	A0_R2	A0_R3	A1_R1	A1_R2	A1_R3	A2_R1	A2_R2	A2_R3	A3_R1	A3_R2	A3_R3
Raw reads	64919028	65615020	65285442	62960278	62869550	64468970	45223700	53167926	53119914	62951976	64892788	63348464
Clean reads	64875898	65574708	65243956	62919044	62825690	64424278	44463942	52093934	52094700	62912590	64847806	63310034
Trinity assembly	257870 transcripts and 223512 genes											
After filter (FPKM > 1)	147570 transcripts and 116545 genes											
After cluster	111390 transcripts and 98514 genes											
GC (%)	42.29											
N50	1368 for transcripts and 1008 for genes											
Genes (FPKM > 5)	16469	14036	15750	15853	15041	13258	16152	14451	14654	15596	13498	15029
Genes (average FPKM > 5)	15414			14658			14963			14849		

**Table 2:** Cold-responsive genes of T. chinensis seeds.

Category	Total	A1 vs. A0^∗^	A2 vs. A0	A3 vs. A0	Shared
Abscisic acid (ABA)	19			0/1	
Aquaporin	22	6/0	2/0	6/0	1/0
C-repeat binding factor (CBF)	3	1/0	1/0	1/0	1/0
Cold stress related	9	0/1			
Cold-regulated protein (COR)	3	0/1			
Heat shock protein (HSP)	36			3/0	
Protein kinase (PK)	529	26/2	16/0	40/13	13/0
Ribosomal protein (RP)	327	5/1		6/1	
Transcription factor (TF)	402	15/25	12/7	31/32	7/5
AP2, AP2-like, AP2/ERF	17	2/0	1/0	3/0	1/0
Ethylene-responsive (ER)	54	5/10	6/5	12/14	3/4
GATA	18	0/3		0/4	
MYB	29	0/3		1/4	
TCP	11			0/1	
WRKY	35	5/2	3/0	4/4	2/0
bHLH	32	0/2		2/2	
bZIP	8	1/0		1/0	
Heat stress	10	1/0	2/0	2/0	1/0
Zinc finger protein (ZFP)	82	7/7	5/2	8/8	3/2
ZAT	17	4/3	5/1	5/4	3/1
Ubiquitin	297	3/3	2/0	6/11	1/0

^∗^Numerator and denominator represent the upregulated and downregulated genes in the comparison.

**Table 3:** Differentially expressed TF genes in *T. chinensis* seeds under cold stress.

Class	GeneID	A1 vs. A0			A2 vs. A0			A3 vs. A0			Description
		Log2FC	FDR	Regulation	Log2FC	FDR	Regulation	Log2FC	FDR	Regulation	
AP2	TR41417|c0_g1	1.65	1.05*E*-03	Up	1.43	1.43*E*-02	Up	1.64	7.33*E*-04	Up	AP2 domain-containing transcription factor family protein
	TR45521|c5_g1	1.20	1.87*E*-02	Up	0.99	1.34*E*-01	NC	1.22	1.09*E*-02	Up	AP2 domain class transcription factor
	TR42026|c0_g1	0.75	2.68*E*-01	NC	0.60	7.29*E*-01	NC	1.12	2.53*E*-02	Up	AP2 domain class transcription factor
ER	TR58370|c0_g1	0.26	8.85*E*-01	NC	0.66	6.05*E*-01	NC	1.63	3.74*E*-04	Up	Ethylene-responsive transcription factor, putative
	TR9006|c0_g1	-1.24	1.44*E*-02	Down	-0.88	2.36*E*-01	NC	-1.12	2.33*E*-02	Down	Ethylene-responsive transcription factor homolog, partial
	TR5872|c0_g1	0.20	9.29*E*-01	NC	-0.04	1.00*E*+00	NC	-1.13	3.50*E*-02	Down	Ethylene-responsive transcription factor ERF118-like
	TR47899|c0_g3	1.19	1.96*E*-02	Up	0.93	1.79*E*-01	NC	1.34	4.16*E*-03	Up	Ethylene-responsive transcription factor ERF118
	TR8021|c0_g1	1.96	1.80*E*-04	NC	1.98	3.72*E*-04	Up	3.45	1.12*E*-12	Up	Ethylene-responsive transcription factor ERF109-like
	TR34720|c0_g2	2.48	1.22*E*-04	NC	3.13	1.10*E*-06	NC	5.29	2.62*E*-21	NC	Ethylene-responsive transcription factor ERF109
	TR43918|c0_g1	1.08	4.21*E*-02	Up	1.01	1.19*E*-01	NC	1.81	5.26*E*-05	Up	Ethylene-responsive transcription factor ERF105-like
	TR44435|c0_g1	-0.18	9.35*E*-01	NC	-0.39	1.00*E*+00	NC	-1.35	3.95*E*-03	Down	Ethylene-responsive transcription factor ERF105
	TR15305|c0_g2	-1.36	5.82*E*-03	Down	-1.21	3.53*E*-02	Down	-2.18	1.19*E*-06	Down	Ethylene-responsive transcription factor ERF096
	TR52068|c0_g1	-0.74	2.68*E*-01	NC	-0.58	7.41*E*-01	NC	-1.81	5.43*E*-05	Down	Ethylene-responsive transcription factor ERF073
	TR78189|c0_g1	-0.76	4.70*E*-01	NC	-0.41	1.00*E*+00	NC	-1.33	4.60*E*-02	Down	Ethylene-responsive transcription factor ERF053
	TR29163|c0_g1	0.90	1.86*E*-01	NC	1.10	1.13*E*-01	NC	1.85	1.09*E*-04	Up	Ethylene-responsive transcription factor ERF023
	TR101055|c0_g1	1.79	5.32*E*-04	NC	1.37	3.22*E*-02	Up	1.51	3.51*E*-03	Up	Ethylene-responsive transcription factor ERF021
	TR15121|c0_g1	-2.77	5.79*E*-08	Down	-1.76	1.33*E*-03	Down	-3.15	6.13*E*-10	Down	Ethylene-responsive transcription factor ERF020
	TR63055|c0_g1	-2.87	4.87*E*-10	Down	-1.50	4.15*E*-03	Down	-2.99	5.23*E*-11	Down	Ethylene-responsive transcription factor ERF020
	TR43748|c0_g2	2.33	3.45*E*-07	Up	1.95	5.74*E*-05	Up	2.73	9.01*E*-10	Up	Ethylene-responsive transcription factor ERF017-like
	TR44877|c0_g1	1.04	7.20*E*-02	Up	1.15	6.95*E*-02	Up	2.17	1.94*E*-06	Up	Ethylene-responsive transcription factor ERF014-like
	TR40856|c0_g1	-1.83	6.38*E*-05	Down	-1.13	5.60*E*-02	Down	-1.22	1.09*E*-02	Down	Ethylene-responsive transcription factor ERF010-like
	TR34995|c0_g1	-1.13	3.80*E*-02	Down	-0.68	5.93*E*-01	NC	-1.13	2.98*E*-02	Down	Ethylene-responsive transcription factor ERF003-like
	TR28226|c0_g1	-1.25	2.08*E*-02	Down	-0.74	5.11*E*-01	NC	-1.34	9.29*E*-03	Down	Ethylene-responsive transcription factor ERF003-like
	TR48171|c0_g1	-0.49	6.08*E*-01	NC	-0.50	8.86*E*-01	NC	-1.15	1.86*E*-02	Down	Ethylene-responsive transcription factor CRF5-like
	TR18144|c0_g1	0.49	6.13*E*-01	NC	0.76	4.22*E*-01	NC	1.67	2.76*E*-04	Up	Ethylene-responsive transcription factor CRF4-like
	TR58185|c0_g1	0.94	1.04*E*-01	NC	1.18	4.33*E*-02	Up	2.30	2.19*E*-07	Up	Ethylene-responsive transcription factor 4-like
	TR47594|c1_g9	1.56	9.17*E*-03	UP	1.53	2.48*E*-02	Up	1.99	2.01*E*-04	Up	Ethylene-responsive transcription factor 3-like
	TR47594|c1_g12	0.97	8.25*E*-02	NC	0.90	2.10*E*-01	NC	1.45	1.65*E*-03	Up	Ethylene-responsive transcription factor 3
	TR32067|c0_g1	-1.15	2.64*E*-02	Down	-0.86	2.67*E*-01	NC	-1.33	4.88*E*-03	Down	Ethylene-responsive transcription factor 2-like
	TR147950|c0_g1	-2.26	6.20*E*-05	Down	-1.59	1.68*E*-02	Down	-3.05	1.90*E*-07	NC	Ethylene-responsive transcription factor 1B
	TR33516|c0_g1	-1.54	3.72*E*-03	Down	-1.11	1.17*E*-01	NC	-2.49	1.17*E*-06	Down	Ethylene-responsive transcription factor 1B
GATA	TR117820|c0_g1	-1.234524683	0.037374327	Down	-0.87	3.95*E*-01	NC	-1.85	4.42*E*-04	Down	GATA transcription factor 4
	TR36890|c0_g1	-1.243857355	0.015695749	Down	-0.95	1.80*E*-01	NC	-1.62	5.01*E*-04	Down	GATA transcription factor 4
	TR44658|c0_g1	-1.202903489	0.020192595	Down	-0.73	4.71*E*-01	NC	-1.00	5.33*E*-02	Down	GATA transcription factor 21 isoform X1
	TR35784|c0_g1	-0.74731694	0.257655438	NC	-0.73	4.62*E*-01	NC	-1.42	2.26*E*-03	Down	GATA transcription factor 1 isoform X2
WRKY	TR40062|c0_g3	-0.215652688	0.914437172	NC	-0.31	1.00*E*+00	NC	-1.20	1.39*E*-02	Down	WRKY8 transcription factor
	TR49705|c0_g1	-1.41602226	0.003732422	Down	-0.85	2.81*E*-01	NC	-0.65	2.91*E*-01	NC	WRKY3 transcription factor
	TR63021|c0_g1	1.964320274	5.63E-05	Up	1.21	6.65*E*-02	Up	1.18	2.83*E*-02	NC	WRKY-type transcription factor
	TR44228|c1_g1	1.754516263	0.000398175	Up	1.91	2.14*E*-04	Up	3.01	5.62*E*-11	Up	WRKY transcription factor 70
	TR49520|c0_g10	0.71637231	0.288662641	NC	0.61	6.76*E*-01	NC	1.06	3.21*E*-02	Up	WRKY transcription factor 7
	TR46552|c0_g1	2.121438235	4.29E-06	Up	1.67	9.78*E*-04	Up	2.32	2.21*E*-07	Up	WRKY transcription factor 51
	TR40322|c0_g1	-0.885288385	0.131822094	NC	-0.76	3.98*E*-01	NC	-1.39	2.76*E*-03	Down	WRKY transcription factor 44
	TR45024|c0_g1	1.178645608	0.02156575	Up	0.78	3.77*E*-01	NC	1.00	4.83*E*-02	Up	WRKY transcription factor 41
	TR36422|c0_g3	1.340014199	0.008307407	Up	0.89	2.61*E*-01	NC	0.93	8.74*E*-02	NC	WRKY transcription factor 33
	TR37159|c0_g1	-0.571132263	0.48525436	NC	-0.53	8.32*E*-01	NC	-1.01	4.85*E*-02	Down	WRKY transcription factor 31
	TR39273|c0_g1	-1.330766726	0.007657745	Down	-0.80	3.58*E*-01	NC	-1.84	5.22*E*-05	Down	WRKY transcription factor 21
bHLH	TR46437|c2_g1	-0.398719573	0.722357889	NC	-0.45	9.81*E*-01	NC	-1.25	8.73*E*-03	Down	Transcription factor bHLH96
	TR46303|c0_g1	0.633841698	0.398045132	NC	0.61	6.85*E*-01	NC	1.60	4.63*E*-04	Up	Transcription factor bHLH47
	TR50792|c4_g15	0.76970154	0.240486872	NC	0.58	7.54*E*-01	NC	1.14	2.13*E*-02	Up	Transcription factor bHLH35-like
	TR45007|c0_g1	-1.162882999	0.023954374	Down	-0.77	3.83*E*-01	NC	-1.20	1.23*E*-02	Down	Transcription factor bHLH147
	TR33541|c0_g1	-1.092396757	0.041192648	Down	-0.67	5.72*E*-01	NC	-0.86	1.13*E*-01	NC	Transcription factor bHLH117
MYB	TR68102|c0_g2	0.509989482	0.679216055	NC	0.27	1.00*E*+00	NC	1.13	4.42*E*-02	Up	Transcription factor MYB44-like
	TR22911|c0_g1	-1.036055197	0.057505766	Down	-0.71	4.93*E*-01	NC	-1.15	1.93*E*-02	Down	Transcription factor MYB44-like
	TR39216|c0_g1	-0.297865259	0.852027342	NC	-0.36	1.00*E*+00	NC	-1.06	3.98*E*-02	Down	Transcription factor MYB12-like
	TR33910|c0_g1	-0.716544213	0.294088684	NC	-0.63	6.36*E*-01	NC	-1.27	7.70*E*-03	Down	R3 MYB transcription factor
	TR44548|c0_g1	-1.310375775	0.009591119	Down	-0.76	4.23*E*-01	NC	-0.71	2.33*E*-01	NC	R2R3-MYB transcription factor
	TR36770|c0_g1	-1.254012729	0.01222635	Down	-0.84	2.87*E*-01	NC	-0.91	8.14*E*-02	NC	R2R3 Myb30 transcription factor
	TR41284|c1_g1	-0.89944911	0.141069891	NC	-0.69	5.58*E*-01	NC	-1.32	7.06*E*-03	Down	MYB family transcription factor APL isoform X2
Other	TR140849|c0_g1	0.210981264	0.947640239	NC	-0.04	1.00*E*+00	NC	-1.09	9.18*E*-02	Down	Transcription factor TCP20-like
	TR42062|c0_g1	2.31068785	1.32E-05	NC	3.07	3.14*E*-09	NC	4.45	4.54*E*-19	Up	Transcription factor perianthia-like isoform X2
	TR33703|c0_g2	-0.406094596	0.731737523	NC	-0.52	8.98*E*-01	NC	-1.17	2.43*E*-02	Down	Transcription factor IBH1
	TR23952|c0_g1	-1.60728151	0.004248943	Down	-0.94	3.10*E*-01	NC	-0.65	3.70*E*-01	NC	Transcription factor HsfA5a
	TR9240|c0_g2	-0.549836404	0.519567814	NC	-1.21	3.78*E*-02	Down	-0.80	1.56*E*-01	NC	Transcription factor HEC2-like
	TR92214|c0_g1	-2.139301951	4.02E-05	Down	-1.27	5.06*E*-02	Down	-2.18	1.61*E*-05	Down	Transcription factor HEC2-like
	TR48713|c0_g1	0.604566309	0.459558903	NC	0.60	7.42*E*-01	NC	1.20	1.60*E*-02	Up	Transcription factor GTE7-like
	TR49896|c0_g1	1.015592988	0.06218293	Up	0.88	2.33*E*-01	NC	1.35	3.79*E*-03	Up	Transcription factor GTE7
	TR78444|c0_g1	0.29647666	0.876314583	NC	0.44	1.00*E*+00	NC	1.08	5.33*E*-02	Up	Transcription factor GT-3b-like
	TR49572|c1_g5	-1.118309909	0.03538728	Down	-0.58	7.54*E*-01	NC	-0.18	8.67*E*-01	NC	Transcription factor family protein
	TR152976|c0_g1	-0.593007991	0.467699069	NC	-0.68	5.69*E*-01	NC	-1.93	2.77*E*-05	Down	Scarecrow-like transcription factor PAT1
	TR38765|c0_g1	0.980757398	0.098741136	NC	0.97	1.93*E*-01	NC	1.54	1.19*E*-03	Up	Nucleolar transcription factor 1 (LOC104416354)
	TR26896|c0_g1	-1.267152582	0.013342976	Down	-0.41	1.00*E*+00	NC	0.58	3.76*E*-01	NC	Nucleolar transcription factor 1
	TR52018|c3_g1	0.511079894	0.60834591	NC	1.09	9.48*E*-02	NC	2.47	4.46*E*-08	Up	NAC transcription factors 36
	TR45153|c0_g1	2.002734024	2.01E-05	Up	1.61	2.13*E*-03	Up	1.60	7.49*E*-04	Up	Heat stress transcription factor A-4b
	TR44136|c1_g1	0.496820818	0.613845686	NC	1.43	8.21*E*-03	Up	3.07	6.23*E*-12	Up	Heat stress transcription factor A-2d isoform X1
	TR22732|c1_g1	1.171958076	0.023399719	Up	0.84	2.91*E*-01	NC	1.08	2.99*E*-02	Up	bZIP transcription factor bZIP16
	TR48040|c0_g1	-1.350723503	0.008908786	Down	-0.74	4.87*E*-01	NC	-0.73	2.40*E*-01	NC	Transcription factor KAN4 isoform X2

## Data Availability

The raw sequencing data can be accessed from the NCBI Sequence Read Archive (SRA) platform (http://trace.ncbi.nlm.nih.gov/Traces/sra/) under the accession number SRA1234084.

## Abbreviations

CBF: C-repeat binding factor
COR: Cold-regulated protein
HSP: Heat shock protein
PK: Protein kinase
RP: Ribosomal protein
TF: Transcription factor
ZFP: Zinc finger protein
KEGG: Kyoto Encyclopedia of Genes and Genomes
COG: Clusters of Orthologous Groups
GO: Gene Ontology
FPKM: Fragments per million reads per kilo base mapped.

## Supplementary Materials

Supplementary Materials Table S1: primer sequences used for the qRT-PCR experiment. Table S2: gene expression profiles of *T. chinensis* seeds treated by cold for 0 h, 12 h, 24 h, and 36 h. Table S3: differentially expressed genes identified in the *T. chinensis* seeds under cold stress.
